The article "Synergistic combination of violacein and azoles that leads to enhanced killing of major human pathogenic dermatophytic fungi Trichophyton rubrum" was retracted in 2017. Reason: compromised peer review.

# Synergistic combination of violacein and azoles that leads to enhanced killing of major human pathogenic dermatophytic fungi *Trichophyton rubrum*

**DOI:** 10.3389/fcimb.2015.00057

**Published:** 2015-08-11

**Authors:** S. Anju, Nishanth S. Kumar, B. Krishnakumar, B. S. Dileep Kumar

**Affiliations:** ^1^Environmental Technology, CSIR-National Institute for Interdisciplinary Science and TechnologyThiruvananthapuram, India; ^2^Agroprocessing and Natural Products Division, CSIR-National Institute for Interdisciplinary Science and TechnologyThiruvananthapuram, India

**Keywords:** azoles, dermatophytosis, *Trichophyton rubrum*, violacein, synergistic

## Abstract

Superficial mycoses caused by dermatophytic fungi such as *Trichophyton rubrum* represent the most common type of worldwide human infection affecting various keratinized tissues in our body such as the skin, hair, and nails, etc. The dermatophytic infection is a significant public health threat due to its persistent nature and high recurrence rates, and thus alternative treatments to cure this fungal infection are urgently required. The present study mainly focused on the synergistic activity of violacein with four azole drugs (ketoconazole, fluconazole, clotrimazole, and itraconazole) against *T. rubrum*. The synergistic antifungal activities of violacein and azoles were measured by checkerboard microdilution and time-kill assays. In our study, combinations of violacein and azoles predominantly recorded synergistic effect (FIC index < 0.5). Significant synergistic value was recorded by the combination of violacein and clotrimazole. Time-kill assay by the combination of MIC concentration of violacein and azoles recorded that the growth of the *T. rubrum* was significantly arrested after 4–12 h of treatment. The combination of violacein and azoles leads to the enhanced inhibition of mycelial growth and conidial germination. Moreover combination enhanced the rate of release of intracellular materials. Morphological changes by SEM analysis were also prominent with the combination. A normal human cell line [Foreskin (FS) normal fibroblast] was used to check the cytotoxicity of violacein. Interestingly violacein recorded no cytotoxicity up to 100 μg/ml. The *in vitro* synergistic effect of violacein and azoles against clinically relevant fungi, *T. rubrum*, is reported here for the first time. Finally, our findings support the potential use of the violacein as an antifungal agent especially against dermatophytic fungi *T. rubrum*.

## Introduction

Antimicrobial resistances (AMR) in superficial fungal infections are a major worldwide public health problem that affects more than 30% of the human population globally (Asticcioli et al., 2008). Among these fungal diseases, dermatophytosis, or tinea, is one of the most frequently encountered human fungal infections. This infection is caused by various dermatophytic fungal species belonging to the *Trichophyton, Microsporum*, or Epidermophyton genera (Soares et al., 2014). Dermatophytosis is a type of superficial fungal infection produced by dermatophytes, a group of keratinophilic fungi that usually infect the keratinized tissues of our body such as nails, skin, and hair, etc. (Baltazar et al., 2013). This infection mainly occurs in immunocompetent and immunocompromised peoples. *Trichophyton rubrum* is the most important causative agent of fungal infections affecting various keratinized tissues (Baltazar et al., 2013). *T. rubrum* mainly affect nails (onychomycosis) a dermatophytosis of high incidence, and it's very rapid evolution may be observed as one of the major indicator of immunodeficiency conditions such as HIV infection and this infection is of significant risk to cancer patients undergoing chemotherapy (Almeida, 2008; Baltazar et al., 2013) and diabetes mellitus patients. In immunodeficient peoples, onychomycosis caused by *T. rubrum* affect entire fingers and toenails (Almeida, 2008; Baltazar et al., 2013), and it is considered the most common and widespread fungal infectious disease worldwide.

The article "Synergistic combination of violacein and azoles that leads to enhanced killing of major human pathogenic dermatophytic fungi Trichophyton rubrum" was retracted in 2017. Reason: compromised peer review.

Infections caused by *T. rubrum* species are very difficult to treat and very few numbers of antifungals available clinically to control this infection (Bitencourt et al., 2013). The azole group of antifungal agents such as ketoconazole and fluconazole have been used for the treatment of various fungal infections especially dermatomycosis (Aala et al., 2010). Azoles are synthetic drugs and although effective, but, because of increased use, azole resistant pathogens have been reported (Mishra and Tiwari, 2011). Furthermore, they are generally known to cause various side effects. Nowadays, the infectious to fungal diseases become more dangerous, and a number of infections become resistant to many classical clinically used antibiotics. Therefore, the continuing efforts to find out new antifungal agents are necessary and urgently needed. Natural products still remained an important source of drug discovery, providing crucial and unmatched chemical diversity. Most of the antimicrobial drugs used today are derived from natural products or natural product scaffolds (Mishra and Tiwari, 2011).

The violacein is a natural purple, blue pigment isolated from various Gram-negative bacteria including *Chromobacterium violaceum, Collimonas* sp., *Duganella* sp., *Iodobacter fluviatile, Janthinobacterium lividum*, and *Microbulbifer* sp. (Wang et al., 2012). Violacein exhibits many biological properties such as broad-spectrum antimicrobial, antiviral, antiprotozoal, and antioxidant activities (Wang et al., 2012), and exerts significant cytotoxicity toward several tumor cell lines (Wang et al., 2012). Moreover violacein recorded antifungal activity especially against chytrid fungus *Batrachochytrium dendrobatidis* which is responsible for the worldwide decline in amphibian populations (Park et al., 2014). Various biological and pharmacological properties of violacein have made it an attractive tool for medical and biotechnological research (Wang et al., 2012).

The article "Synergistic combination of violacein and azoles that leads to enhanced killing of major human pathogenic dermatophytic fungi Trichophyton rubrum" was retracted in 2017. Reason: compromised peer review.

For several years until now, combination therapy with two or more antibiotics is used to prevent or delay the emergence of drug-resistant strain to take advantage of antibiotic synergism (Chambers, 2006). Recently, the combinations of natural products and antibiotics were reported to enhance the activity of classical antibiotics (Reuk-ngam et al., 2014). Thus, the synergistic interactions of natural products and standard antibiotics were a potential alternative approach to treating various infectious diseases. In the view of our ongoing research for promising antimicrobial agents and explore the novel biological activity of violacein, we decided to study the synergistic effects of violacein with four classical antifungal agents with special reference to human pathogenic fungi *T. rubrum*.

## Materials and methods

### Violacein

Violacein (Figure 1) used in the present study was isolated from a novel strain of *Chromobacterium violaceium* isolated from sediment sample collected from a clay mine acid lake in Thiruvananthapuram district in Kerala, India (Lat_long = 8°5553″ N 76°8577″E). The culture was maintained in 0.1% peptone water media (0.01 g peptone, 0.003 g NaCl/10 ml distilled water) in room temperature in small vials. It was sub-cultured bimonthly. After 24 h fermentation in LB broth, the bacterial biomass was separated through centrifugation the biomass was extracted twice with ethanol. The ethanolic extract was filtered through 0.22 μm filter paper (Millipore) to avoid the cell detritus and then dried in the rotavapour. The pure violacein was precipitated by methanol water crystallization and then the precipitate was washed with hexane and demineralized water. Violacein obtained was then dried in an oven at 80°C and kept in a desiccator and its structure was confirmed by the spectroscopic methods (^1^H NMR and MS).

**Figure 1:** **Chemical structure of violacein and azoles used in the present study**. Violacein were isolated and purified from a novel strain of *Chromobacterium violaceum* and azoles drugs were purchased from Sigma-Aldrich.

The article "Synergistic combination of violacein and azoles that leads to enhanced killing of major human pathogenic dermatophytic fungi Trichophyton rubrum" was retracted in 2017. Reason: compromised peer review.

### Azole agents

Ketoconazole, fluconazole, clotrimazole, and itraconazole (Figure 1) were used as standard antifungal agents and were purchased from Sigma Chemical Co. (St Louis, MO). Antifungal agents were prepared as stock solutions at concentrations of 2 mg/ml in dimethylsulfoxide for susceptibility testing and checkerboard method, respectively.

### Test pathogens

The test dermatophyte *T. rubrum* (MTCC 296) was procured from Microbial Type Culture Collection and Gene Bank (MTCC) Division, CSIR-Institute of Microbial Technology (IMTECH), Chandigarh, India. The strains were cultivated on Potato dextrose agar (PDA) (Hi-media, Mumbai, India) and incubated at 28°C for 7–15 days. For all experiments, the strains were cultivated on PDA and incubated at 28°C as described above or until the sporulation.

### Preparation of inoculum

*T. rubrum* colonies were covered with 5 ml of sterile saline solution (0.85%), the surface was gently scraped using a sterile inoculating loop and the saline solution with fungal materials was gently transferred to a sterile test tube. This suspension was shaken for 2–3 min using a vortex mixer, allowed to stand for 5 min to allow hyphal fragments to fall out of the suspensions so that the supernatant containing the conidia could be collected. Inocula were standardized at 0.5 tube of McFarland scale (10^5^ CFU/ml). Quantification was confirmed by inoculating 0.01 ml of a 1:100 dilution of each suspension onto PDA. The PDA plates were incubated at 28°C and the developments of fungal colonies were examined daily.

### Determination of minimum inhibitory concentration (MIC)

The MIC value of violacein and azole antibiotics were performed using the microdilution assay as described in M38-A2, Clinical and Laboratory Standards Institute (CLSI, 2008), with minor modifications. The medium used was RPMI 1640 with L-glutamine (Sigma-Aldrich, St. Louis, MO, USA) buffered to pH 7.0 with 0.165 M morpholine propanesulfonic acid (MOPS) (Sigma-Aldrich, USA), supplemented with 2% glucose. The *T. rubrum* cell suspension was prepared in a 0.85% saline solution. The suspension of conidia was then transferred to sterile test tubes where they remained for 30 min to separate the microconidia, which were lighter and therefore, present in the supernatant. After that the separated microconidia concentration was adjusted to obtain a final concentration ranging from 3 × 10^3^ to 6 × 10^3^ CFU/ml. Then these suspensions were diluted in RPMI 1640 (Sigma-Aldrich, St. Louis, MO, USA) and inoculated on 96-well plates that had been previously prepared with the test compounds diluted at concentrations from 0.5 to 1000 μg/ml. Positive (medium with inoculum) and negative (medium alone) controls were included in all experiments. The plates were incubated for 7 days at 28°C. The MIC reading was performed by spectrophotometry at 600 nm. The MIC was defined as the concentration of violacein/azoles that inhibit 90% of fungal growth.

The article "Synergistic combination of violacein and azoles that leads to enhanced killing of major human pathogenic dermatophytic fungi Trichophyton rubrum" was retracted in 2017. Reason: compromised peer review.

### Minimum fungicide concentration (MFC)

Aliquot of 20 μl from the wells that recorded no fungal growth in MIC test was serially diluted and plated on a PDA plates and incubated at 28°C for 5 days. The MFC was defined as the lowest violacein/azoles concentration that did not allow the growth of any fungal colonies on the PDA plates after the incubation period (Soares et al., 2014).

### Synergistic effect of violacein and azoles

The drug interaction activity was assessed using a checkerboard method derived from a standardized procedure recommended by the Clinical and Laboratory Standards Institute (M38-A2) (CLSI, 2008). Briefly, the test was performed in the same medium used for susceptibility testing. Volumes of 150 μl of the MIC concentration of violacein and azoles were dispensed in 96-well plates. To each well, 50 μl of the fungal suspension was added to produce a final concentration of 5 × 10^3^ CFU/ml. The negative control contains 200 μl of RPMI while the positive control contains 150 μl of RPMI medium with 50 μl of inoculum. The plates were incubated at 28°C, and the reading was completed after 5 days. We conducted visual and spectrophotometric readings at 600 nm. To determine the effect of combinatorial fractions, we calculated the fractional inhibitory concentration (FIC). The FIC was calculated by taking the MIC of the compound in combination/MIC of the compound alone. The sum of the fractional inhibitory concentration (FIC) of each compound consists of the fractional inhibitory concentration index: (The MIC of compound A in combination/The MIC of compound A alone) + (The MIC of compound B in combination/The MIC of compound B alone). A synergistic relationship was defined as FIC index ≤ 0.5, an additive relationship was defined as 0.5 < FIC index ≤ 1.0, an indifferent relationship was defined as 1.0 < FIC index ≤ 4.0, and an antagonistic relationship was defined as FIC index >4.0 (Soares et al., 2014).

### Time–kill studies

The time–kill activity was determined to know the rate of killing of *T. rubrum* conidia. A time–kill curve (CFU as a function of time) is evaluated to study the rate and extent of reduction in *T. rubrum* conidia when treated with violacein and azoles individually and in combination. The time–kill was conducted for 48 h in Potato Dextrose Broth (PDB). The concentrations used are the MIC values of violacein and azole drugs alone and in combination (see Table 1). An initial inoculum of approximately 1 × 10^6^ CFU/ ml conidia was taken for all the experiments. At predetermined time points (0, 2, 4, 6, 8, 12, 24, and 48 h), a 0.1 ml sample was removed and serially diluted in normal saline and plated onto PDA plates. Colony counts were determined following 5 days of incubation at 30°C. The broth without any test compounds was used as the control. The data were plotted as log CFU/ml vs. time (h) for each time point. Tests were performed in triplicate (Khan and Ahmad, 2011).

The article "Synergistic combination of violacein and azoles that leads to enhanced killing of major human pathogenic dermatophytic fungi Trichophyton rubrum" was retracted in 2017. Reason: compromised peer review.

**Table 1:** **Synergistic effects of the violacein in combination with azole drugs against *T. rubrum***.

**Test organism**	**Agent**	**MIC/MFC (μg/ml)**		**FIC/FFC**	**FICI^b^/FFCI^c^**	**Outcome**
		**Alone**	**Combination^a^**			
*T. rubrum*	Violacein Ketaconazole	32/64 1/2	2/4 0.25/0.25	0.06/0.06 0.13/0.13	0.19/0.19	Synergistic/synergistic
	Violacein Fluconazole	32/64 2/4	4/4 0.5/0.5	0.13/0.06 0.25/0.13	0.38/0.19	Synergistic/synergistic
	**Violacein** **Clotrimazole**	**32/64** **4/8**	**1/2** **0.25/0.25**	**0.03/0.03** **0.06/0.03**	**0.09/0.09**	**Synergistic/synergistic**
	Violacein Itraconazole	32/64 2/2	8/8 0.25/0.5	0.25/0.13 0.13/0.25	0.38/0.38	Synergistic/synergistic

*MIC/MFC value of violacein and azoles alone was conducted by micro broth dilution method and MIC/MFC value of the combination was conducted by checkerboard assay. FICI index were obtained from the checkerboard assay: To evaluate the interaction of violacein with azoles against T. rubrum, checkerboard experiments were performed. FIC/FFC index = (MIC/MFC of azoles in combination with violacein/MIC/MFC of azoles alone) + (MIC/MFC of violacein in combination with azoles/MIC/MFC of violacein alone). A FICI/FFCI ≤ 0.5 is indicative of synergism*.

a *The MIC and MFC of violacein in combination with azole*.

b *The fractional inhibitory concentration index (FIC index)*.

c *The fractional fungicidal concentration index (FBC index)*.

*Values in bold indicated best synergistic combination*.

### Effects of the combination on mycelial growth

Analysis of the influence of violacein and azole drugs on mycelial growth was studied by assessing the mycelial dry weight of *T. rubrum* in triplicate (Pereira et al., 2013). PDB (5 ml) with violacein and azoles individually and in combination and 0.5 ml of the inoculum suspension were added to sterile tubes. Control tubes involved the use of sterile distilled water in place of the test compounds. The tubes were incubated at 28°C for 10 days, the mycelia filtered through sterile filter paper (retention of particles: 10 μm) and then dried at 50°C for 15–20 min. The filter paper containing dry mycelia was weighed, and the percent of mycelia produced was calculated, using the growth in the control tubes as being 100% of potentially dry mycelial weight.

The article "Synergistic combination of violacein and azoles that leads to enhanced killing of major human pathogenic dermatophytic fungi Trichophyton rubrum" was retracted in 2017. Reason: compromised peer review.

### Effects of the combination on conidial germination

Violacein and azoles were tested to evaluate their impact on the germination of *T. rubrum* conidia. Double concentrated PDB (1 ml) containing the violacein and azoles individually and in combination was added to sterile tubes, mixed with 500 μl of fungal suspension and then immediately incubated at 28°C. Samples were taken at 24 h to record the number of germinated and ungerminated conidia through the use of a hemocytometer from which the percentage of germinated conidia was calculated. The test was conducted in triplicate (Pereira et al., 2015).

### Effect of combination on the release of intracellular material

Measurements of the release of fungal intracellular material absorbing at 260 nm from *T. rubrum* were conducted using 5 ml aliquots of the fungal inocula after the addition of the violacein and azoles alone and in combination. At different time intervals (2, 4, and 6 h), fungal cells were centrifuged at 5000 rpm for 5 min, and the supernatant was examined by measuring the absorbance at 260 nm with a UV-visible spectrophotometer (Shimadzu). The flask without test violacein and azoles was used as the control. Alcoholic potassium hydroxide solution (25% diluted with ethanol at 70%) was used as the reference compound since it causes 100% cellular leakage. Rate of release of intracellular material absorbing at 260 nm, primarily nucleotides, was calculated by comparing the test values with the lysing agent which was considered to be 100%. The experiment was performed in triplicate (Pereira et al., 2013).

### Morphological studies by scanning electron microscope (SEM)

The plates used for studying the antifungal activity by disc diffusion were employed in the morphological studies using SEM. Samples of mycelial growth were taken at the central, intermediate, and peripheral zones of the colonies. SEM analysis of adhesive tapes used to capture fungal structures was made using a SEM (JEOL JSM 5600 LV Electron Microscopy (USA). Tape fragments measuring 5–10 mm in diameter bearing the fungal structures were cut and mounted onto a 12 mm metal stub (Agar Scientific, Essex, England, pin stubs cod. G301F), using double-sided carbon adhesive tape. The morphological characteristics of the hyphae, conidiophores, phialides, spores, and conidia were determined with SEM analysis (Michaelsen et al., 2010).

### Cytotoxicity test by MTT assay

The MTT (3-(4, 5-dimethyl thiazol-2-yl)-2, 5-diphenyl tetrazolium bromide) (Sigma-Aldrich) assay was employed to determine the toxicity of violacein against FS (Foreskin) normal fibroblast cell line, a normal human cells line (Anto et al., 2003; Kumar et al., 2014).

The article "Synergistic combination of violacein and azoles that leads to enhanced killing of major human pathogenic dermatophytic fungi Trichophyton rubrum" was retracted in 2017. Reason: compromised peer review.

### Statistical analyses

The statistical analyses were performed with SPSS (Version 17.0; SPSS, Inc., Chicago, IL, USA). In the case of MIC, MFC, and FICI experiments, when the results were different in both experiments, we made another test for the final result. For time-kill assay, One-Way ANOVA (Duncan's multiple range) tests was used and the data was presented as means ± standard deviations. Statistical significance of the experiments was defined as *p* < 0.05.

## Results

### MIC and MFC

MIC and MFC value of violacein and four azole antibiotics used alone for *T. rubrum* are shown in Table 1. The MIC/MFC value of violacein against *T. rubrum* was 32/64 μg/ml. The MIC/MFC values of azole drugs ranges from 1 to 8 μg/ml, and the highest activity was recorded by ketoconazole 1 μg/ml (Table 1).

### Synergistic effect by checkerboard assay

The synergistic activities of violacein and azole drugs from the checkerboard assay against the *T. rubrum* are shown in Table 1. FIC, FFC, FIC index, FFC index, and interpretations for the activities of violacein and azole drugs against the *T. rubrum* predominantly recorded the synergistic interaction. A best synergistic interaction was recorded by the combination of violacein and clotrimazole (Table 1).

### Time-kill assay

The time-kill assay of violacein and azoles alone and in combination is shown in Figure 2. The combination of violacein and azole drugs recorded significant reduction in the CFU/ml when compared to the effect of individual compounds (violacein and azoles) (Figure 2). For the combination of violacein and ketoconazole, the significant reduction in the CFU/ml was recorded between 6 and 12 h, whereas for violacein and fluconazole it was between 12 and 24 h. The combination of violacein and clotrimazole recorded best reduction in the colony count between 4 and 12 h. But the significant reduction in the colony count was recorded by violacein and itraconazole (4–6 h).

**Figure 2:** **Time–kill curves of violacein and azoles alone and in combination against *T*. *rubrum***. The experiments were performed in triplicates. Data are expressed as mean ± standard deviation. CFU-Colony Forming Unit.  Control,  Violacein,  Azole,  MIC combination,  Half MIC combination.

### Effects combination of violacein and azoles on mycelial growth

The impact of the combination of violacein and azole drugs on the growth of mycelia was determined by measuring the mycelial dry weight of *T. rubrum* after treatment (Figure 3). As shown in Figure 3, the combination of violacein and azoles recorded significant inhibition of the mycelial growth of *T. rubrum* (*P* < 0.05) as compared with that of individual compounds (100% mycelia yield) and control. Best inhibition was recorded by the combination of violacein and clotrimazole (Figure 3).

The article "Synergistic combination of violacein and azoles that leads to enhanced killing of major human pathogenic dermatophytic fungi Trichophyton rubrum" was retracted in 2017. Reason: compromised peer review.

**Figure 3:** **Percentage of dry mycelial weight produced by *T. rubrum* by the treatment of violacein and four azoles alone and in combination**. Control produced 100% of dry mycelial weight. Data are expressed as mean ± standard deviation. Different letters in the superscript were significantly different according to Duncan's multiple range test (*p* < 0.05).

### Effect of combination on the conidial germination

The percentage of germinated conidia of *T. rubrum* after the treatment is recorded in Figure 4. The combination of violacein and azole drugs significantly inhibited conidial germination (*P* < 0.05). Here also best inhibition was recorded by the combination of violacein and clotrimazole (Figure 4).

**Figure 4:** **Percentage of germinated conidia of *T. rubrum* by the treatment of violacein and four azoles alone and in combination**. Data are expressed as mean ± standard deviation. Different letters in the superscript were significantly different according to Duncan's multiple range test (*p* < 0.05).

### Effect of combination on the release of intracellular materials

The effect of violacein and azoles alone and in combination on cell membrane and resulting impact on the release of intracellular materials was initially determined by measurement of the release of 260 nm absorbing intracellular material from *T. rubrum* (Figure 5). From the results, it is clear that the combination of violacein and azoles leads to an enhanced release of intracellular materials from the cell compared to compounds alone and control (no compounds) (*P* < 0.05). Release of intracellular materials starts from 2 h onwards and reached maximum at 4 h and then remain stable (Figure 5)

**Figure 5:** **Rate of release of intracellular material of *T. rubrum* recorded absorbance at 260 nm in the absence (control) and presence of violacein/azoles alone and in combination**. Data are expressed as mean ± standard deviation. Different letters in the superscript were significantly different according to Duncan's multiple range test (*p* < 0.05).

### Morphological changes induced by the combination of violacein and azoles as revealed by SEM analysis

SEM analysis of the morphological changes induced by violacein and azoles revealed that the combination recorded significant morphological changes in *T. rubrum*. Enhanced hyphal damages and rupture were observed with the combination as compared with that of individual compounds (Figure 6). Combinations treated hyphae also recorded wrinkling of the cell surface and emptying of the cytoplasmic content, which were not observed on the smooth surfaces of untreated hyphae. Moreover, the combination enhances severe damaged shown as collapse and degradation of the cells. Drastic reduction of *T. rubrum* spores number was also observed for the combination of violacein and azoles (Figure 6), although to a lesser extent with ketoconazole and fluconazole.

The article "Synergistic combination of violacein and azoles that leads to enhanced killing of major human pathogenic dermatophytic fungi Trichophyton rubrum" was retracted in 2017. Reason: compromised peer review.

**Figure 6:** **Morphological analysis by SEM after the treatment of *T. rubrum* by violacein alone and in combination with azole drugs**. **(A)** control, **(B)** violacein alone, **(C)** violacein +ketoconazole, **(D)** violacein +fluconazole, **(E)** violacein +clotrimazole, and **(F)** violacein +itraconazole.

### Cytotoxicity assay of violacein

The cytotoxic activity of violacein was confirmed using MTT assay against the FS normal fibroblast cell line. The present results clearly showed that violacein recorded no significant cytotoxicity up to 100 μg/ml (Figure 7). The data from MTT assay clearly indicates that violacein may be safe against normal human cells.

**Figure 7:** **Cytotoxicity of violacein against normal human cell line (Foreskin normal fibroblast) conducted by MTT (3-(4, 5-dimethyl thiazol-2-yl)-2, 5- diphenyl tetrazolium bromide) assay**. All measurements were taken in replicates of three, and results are expressed as arithmetic mean ± standard error of the mean. **(A)** Bar diagram of the result at different concentration and **(B)** representative confocal microscopic image of cells.

## Discussion

The novel development of strategies to manage various pathogenic fungal infections may be an effective means for ideal therapeutic interventions. Consequently, the aim of novel antifungal strategies is to develop new drugs that combine sustainability, high efficiency, relatively low toxicity, safe for human beings, animals, plants, and environment with comparatively low production cost. Human pathogenic fungal infections are more prevalent in both developed and developing nations (Cronin et al., 2014). According to World Health Organization (WHO) more than 25% of the global populations are infected with various dermatophytes (pathogenic fungi affecting keratinized materials of our body) (Cronin et al., 2014). Unlike human pathogenic bacteria, fungi are eukaryotic organisms and the treatment to control these become more limited due to the biochemical similarities between human and fungal cells. In addition, treatment becomes more difficult due to the position of infecting area especially beneath the nail and this makes it difficult to administer therapeutic doses of various topical therapies (Seebacher et al., 2008; Cronin et al., 2014). Thus, superficial fungal infections of keratinized tissue and mucous membranes caused by pathogenic dermatophytes become one of the challenging fungal infections to treat. The main therapies currently available to treat dermatophytic fungi have concerns either due to their poor response to the reappearance of infection reported in up to 40% of cases. Moreover the treatment of this fungal infections require high treatment costs, comprehensive treatment requirements and severe side effects (e.g., hepatotoxicity) (Woodfolk, 2005; Warshaw, 2006; Chang et al., 2007). The profound impact dermatophytes have on a patient's quality of life due to the severe pain and physical deformation caused by the infection surely warrants alternative drug that are safe and more effective (Szepietowski and Reich, 2009). Due to the very high rate of recurrence of superficial fungal infections and the increasing antifungal resistance problems, in particular against the azoles, new drugs alternatives with fungicidal activity are very much needed (Ghannoum et al., 2013; Tchernev et al., 2013). In this background, the antifungal activity of violacein against *T. rubrum*, one of the major human pathogenic dermatophytes was evaluated on their own or in combination with four major clinically used azole drugs.

The article "Synergistic combination of violacein and azoles that leads to enhanced killing of major human pathogenic dermatophytic fungi Trichophyton rubrum" was retracted in 2017. Reason: compromised peer review.

An alternative approach to combat drug-resistant fungal pathogens is the use of antifungal agents in combination with natural compounds to reduce toxicity and the emergence of multidrug resistance (Endo et al., 2010). In view of the lack of novel drugs with different molecular targets and mechanism of action, combination of two or more drug might be considered as a viable strategy for therapy, considering the multiplicity of fungal targets against which current agents are effective (Mukherjee et al., 2005; Endo et al., 2010). The combinations of the drug are described as synergy, indifferent, additive or antagonistic. The main benefit of using drug combination is the synergistic effect, in which the activity is greater than the individual drugs (Endo et al., 2010). In current study violacein and azole combination recorded activity at very low concentration than the individual compounds. The benefits of using synergistic drug combination include a wider spectrum of efficiency, improved safety and tolerability and an enhanced reduction of antifungal resistance (Lewis and Kontoyiannis, 2001; Endo et al., 2010). In our study, we investigated the synergistic effect of violacein and four clinically used azole drugs (ketoconazole, fluconazole, itraconazole, and clotrimazole). We mainly focused on the combinations of violacein with azoles because azole is one of the most accepted antifungal agent used for treating dermatophytes, especially in patients with the immunocompromised condition.

The article "Synergistic combination of violacein and azoles that leads to enhanced killing of major human pathogenic dermatophytic fungi Trichophyton rubrum" was retracted in 2017. Reason: compromised peer review.

In our study, significant synergy was recorded by violacein in combination with azole antibiotics. This is in agreement with the earlier studies that the efficacy of azole drugs can be improved by certain natural products (Aala et al., 2010; Endo et al., 2010). Violacein used in our study was a natural product predominantly isolated from *Chromobacterium* spp. and this compound significantly enhanced the activity the four azole drugs employed in the current study. Positive interactions in checkerboard microdilution were confirmed by time-killing assay. Time-kill curves can provide growth kinetic information over time. This method is often used to detect the differences in the rate and extent of antifungal activity over time (Jin et al., 2010). In the present study, there was an excellent agreement between the FICI method and the time-kill curves. The combination of violacein and azole drugs recorded significant synergistic interaction against *T. rubrum*. Thus, the combination of violacein with azole drugs represents an attractive alternate approach for the development of new management strategies for controlling superficial dermatophytic infections. Previously the synergistic antibacterial activities of violacein with antibiotics are reported (Subramaniam et al., 2014). Moreover, the synergistic effect of violacein and azoles against medically important dermatophytic fungi like *T. rubrum* is reported here for the first time.

In case of dermatophytosis pathogenesis, dermatophytes produce filamentous hyphae during the infection process in our body. It is important because they can exacerbate the damage and penetrate into the deeper layers keratinized tissues of our body (Pereira et al., 2015). Therefore, the dry mycelial mass does not reflect the total live cells, but equally important, it reflects the production of the fungal cell material. In the present study, the combination of violacein and azoles inhibited the fungal growth by decreasing the dry mycelial production of *T. rubrum*. So the present study clearly demonstrated that the combination will help to control the growth of fungal hyphae and thus prevent the occurrence of infections in deeper layers of our body.

*T. rubrum* conidia are considered as one of the primary means of establishing dermatophytosis in humans and animals. They adhere to epithelial cells of the keratinized tissues of the host where they germinate and initiate an invasion of the stratum corneum. Hyphae can grow in multiple directions and form mycelium (Ohara and Tsuge, 2004). The findings of the present study clearly demonstrated that the combination of violacein and azoles inhibited the germination of conidia, and this is of particular significance that this will prevent the further dissemination of *T. rubrum*.

The article "Synergistic combination of violacein and azoles that leads to enhanced killing of major human pathogenic dermatophytic fungi Trichophyton rubrum" was retracted in 2017. Reason: compromised peer review.

Ergosterol is a sterol found in the cell membranes of yeasts and filamentous fungi and functions as an important regulator of membrane fluidity. Changes in the ergosterol biosynthetic pathway will also inhibit fungal growth (Van Minnebruggen et al., 2010). The azoles mainly act through the inhibition of lanosterol-14a-demethylase, a key enzyme involved in the biosynthesis of ergosterol, an important component of the fungal cell membrane (Martinez-Rossi et al., 2008). In *T. rubrum*, azoles treatment significantly reduces the ergosterol level within the cell, leading to the cell membrane perturbation. The azole portion in the combination decreases the sterol concentration which in turn leads to cell membrane perturbation (Uppuluri et al., 2008). The resulted in the alteration of plasma membrane permeability that allows violacein portion in the combination to enter the cell and that may lead to the enhanced killing of *T. rubrum*. The proposed mechanism of action of the synergistic combination of violacein and azole is shown in Figure 8. Because of these effects on fungal membranes, we investigated whether violacein and azole alone and in combination damages the cell membrane of *T. rubrum* by the detection of intracellular components released into the external environment. These cellular components represent primarily nucleotides, and that recorded strong absorption at 260 nm. Our results clearly suggest that violacein azole combination interferes with the integrity of the cell membrane producing damage to the structure. We also speculate that resulting alterations in the plasma membrane permeability may allow increased concentrations of violacein to enter the cell, resulting in enhanced fungal cell death. Moreover, azoles reduce the sterol concentration in fungal cells and, thereby, its combination with violacein renders the combination fungicidal. In future research based on *T. rubrum* infected animal models may resolve the *in vivo* efficacy of the synergistic combination violacein and azoles.

**Figure 8:** **Proposed mechanism of action of the synergistic combination of violacein and azoles**. Where “V” denotes violacein and “A” denotes azole drugs.

The significant biological and pharmacological activities of violacein have made it an attractive area for many medical researchers. It is reported that intraperitoneal doses of violacein up to 1 mg/kg are not toxic in mouse blood, kidneys, or liver, which provides evidence for the *in vivo* use of violacein as a therapeutic agent with little side effects (Cazoto et al., 2011). In the present also violacein was non-toxic to a normal healthy human cell line (FS) up to 100 μg/ml.

The article "Synergistic combination of violacein and azoles that leads to enhanced killing of major human pathogenic dermatophytic fungi Trichophyton rubrum" was retracted in 2017. Reason: compromised peer review.

## Conclusions

In our study, violacein exhibited significant antifungal activity, and this proved its efficacy as potential antifungal agent. Interestingly violacein exhibited strong synergistic interactions with azole drugs against the *T. rubrum*. These results suggest that the combination of violacein and azoles can be expected to act synergistically in the treatment of dermatophytic infections. Further investigation is required to examine the effects of violacein and azoles combination against other clinically relevant dermatophytes. The current studies also draw attention for developing new compounds from natural source especially violacein as antifungal agents in the management of dermatophytosis. However, *in vivo* experimental evaluations are needed to unfold the therapeutic potential of these agents in combating such superficial fungal diseases.

### Conflict of interest statement

The authors declare that the research was conducted in the absence of any commercial or financial relationships that could be construed as a potential conflict of interest.
